# MicroRNA-613 inhibits cell growth, migration and invasion of papillary thyroid carcinoma by regulating SphK2

This article has been retracted.

**DOI:** 10.18632/oncotarget.9530

**Published:** 2016-05-21

**Authors:** Wangwang Qiu, Zhili Yang, Youben Fan, Qi Zheng

**Affiliations:** ^1^ Department of General Surgery, Shanghai Jiao Tong University Affiliated Sixth People's Hospital, Shanghai 200233, P.R. China

**Keywords:** papillary thyroid cancer, miR-613, SphK2, cell growth, invasion

## Abstract

MicroRNAs (miRNAs) have emerged as important gene regulators and are recognized as key players in carcinogenesis. In this study, we investigated the biological function and mechanism of miR-613 in the regulation of papillary thyroid cancer (PTC) development. We found that miR-613 was downregulated in PTC cell lines and tissues, and overexpression of miR-613 significantly suppressed PTC cell growth, migration and invasion *in vitro* and inhibited tumor growth *in vivo*. We identified the gene for sphingosine kinase 2 (*SphK2*) as a direct target of miR-613. Overexpression of miR-613 significantly repressed SphK2 expression by directly targeting its 3′-untranslated regions (3′-UTR) and restoration of SphK2 reversed the inhibitory effects of miR-613 on PTC cell growth and invasion. Taken together, our results indicated that miR-613 functions as a tumor suppressor in PTC and its suppressive effect is mediated by repressing SphK2 expression.

## INTRODUCTION

Thyroid cancer is one of the few malignancies that are increasing in incidence in the world [1, 2]. Thyroid cancer is classified into four types: papillary, follicular, medullary, and anaplastic thyroid cancer. Papillary thyroid cancer (PTC) is the most common type, accounting for greater than 80% of all thyroid cancers, and is a major type mainly in young women and children [3, 4]. Understanding the molecular mechanism of the proliferation, migration, and invasion of PTC is important for the development of more effective therapeutic strategies.

MicroRNAs (miRNAs) are small, endogenous, noncoding RNAs of approximately 22 nt that regulate the expression of target mRNA by binding to 3′-untranslated regions (UTRs), resulting in target mRNA degradation or silencing [5, 6]. Aberrant expression of miRNAs can act as tumor suppressors or oncogenes, depending on the cellular function of their targets [7, 8]. Several studies suggest that alterations in miRNA expression contribute to PTC development and progression [9–13]. In our previous study, miRNA-613 was significantly downregulated in PTC tissues compared with adjacent non tumor tissues by miRNA arrays and qRT-PCR analysis [14]. However, no evidence of miR-613 function in PTC has been documented.

Sphingolipids are a diverse group of water-insoluble molecules that includes ceramides, sphingoid bases, ceramide phosphates and sphingoid-based phosphates [15]. The dynamic balance of ceramide phosphates and sphingoid-based phosphates determines cell proliferation, invasion and apoptosis [16]. Sphingosine kinases (SphKs) are the main limiting enzymes for sphingoid-base phosphates in cells and have two distinct isoforms, Sphk1 and SphK2 [17, 18]. SphK1, an oncogenic kinase, is elevated in various human cancer types and is involved in tumor development and progression including in thyroid cancer [19]. The biological functions of SphK2 in thyroid cancer remain unknown.

In this study, we verified miR-613 downregulation in PTC cell lines and tissues. We found that miR-613 overexpression significantly inhibited cell proliferation, migration and invasion by targeting SphK2 *in vitro* and suppressed tumor growth *in vivo*. Our study demonstrated that miRNA-613 negatively regulates SphK2 and is involved in proliferation and invasion-related processes in PTC.

## RESULTS

### MiR-613 is frequently downregulated in PTC

We investigated the expression of miR-613 in three PTC cell lines (TPC-1, BCPAP and K1), using the human thyroid epithelial cell line Nthy-ori3-1 as a control. We found that miR-613 was downregulated in PTC cell lines compared with the human thyroid epithelial cell line (Figure 1A). We also examined miR-613 expression in 20 pairs of PTC tissue specimens and adjacent nontumor tissues. The results showed that miR-613 expression was significantly decreased in PTC tissues compared with paired adjacent nontumor tissues (Figure 1B). These results indicated that low miR-613 might be associated with PTC development.

**Figure 1:** miR-613 is downregulated in PTC cell lines and patient specimens (**A**) miR-613 was detected in PTC cell lines and normal thyroid cells using qRT-PCR. (**B**) Expression of miR-613 was measured in 20 pairs of PTC tissue specimens (**C**) and adjacent nontumor thyroid tissues (N) using qRT-PCR. Each sample was tested three times.*P < 0.05.

### MiR-613 inhibits cell growth, invasion and migration *in vitro*

To explore the possible biological functions of miR-613 in PTC cells, we transfected K1 and TPC-1 cell lines with miR-613 mimics or negative controls. MTT assays demonstrated that miR-613 overexpression significantly inhibited PTC cell proliferation compared with negative control cells (Figure 2A). We also examined the colony formation capacity of K1 and TPC-1 cells. The results suggested that PTC cells formed fewer colonies when infected with miR-613 lentivirus compared with control groups (Figure 2B). To investigate the effect of miR-613 on cellular motility, we used transwell assays to measure the migration and invasion ability of K1 and TPC-1 cells after modification of miR-613 expression. Cells migrating through the transwell were reduced in miR-613-transfected K1 and TPC-1 cells (Figure 2C). Similarly, invasive cells were decreased in miR-613-transfected cells (Figure 2D). We next examined the effects of miR-613 loss of function on PTC cell proliferation, migration and invasion. BCPAP cells were transfected with miR-613 inhibitor (anti-miR-613) or control miRNA (anti-miR-C). As expected, inhibition of miR-613 significantly promoted cell proliferation, migration and invasion in BCPAP cells when compared with negative control cells (Supplementary Figure S1). Collectively, these results indicated that miR-613 may impede cellular proliferation, cell migration and invasion *in vitro*.

**Figure 2:** Overexpression of miR-613 suppresses proliferation, migration and invasion of K1 and TPC-1 cells (**A**) Cell viability was determined by MTT assays on K1 and TPC-1 cells transfected with miR-613 mimics or negative control. (**B**) K1 and TPC-1 cells were transduced with miR-613 lentivirus or negative controls for colony formation assays. (**C**–**D**) Transwell migration and Matrigel invasion assays on K1 and TPC-1 cells transfected with miR-613 mimics or negative control. *P < 0.05.

### MiR-613 inhibits tumor growth of PTC *in vivo*

We investigated whether ectopic expression of miR-613 repressed tumor growth *in vivo*. TPC-1 cells transduced with Lv-miR-613 or Lv-ctrl were subcutaneously injected into nude mice. After 36 days, mice were killed and miR-613 expression was measured. MiR-613 expression was higher in the Lv-miR-613 group than in the Lv-ctrl group (Figure 3A). Tumors overexpressing miR-613 grew more slowly and were smaller than control tumors (Figure 3B–3C). An approximately 2.5-fold decrease in tumor weight was observed in miR-613-overexpressing tumors compared to controls (Figure 3D). These results suggested that miR-613 inhibited PTC cell growth *in vivo*.

**Figure 3:** miR-613 inhibits PTC cell growth *in vivo* TPC-1 cells were infected with Lv-miR-613 and injected subcutaneously into nude mice. (**A**) Expression of miR-613 in xenograft tumorswas determined by qRT-PCR. (**B**) Growth curve of tumor volumes. (**C**) Representative photograph of xenograft tumors. (**D**) Tumor weight. *P < 0.05.

### SphK2 is the target of miR-613

To investigate the mechanism by which miR-613 suppresses PTC cell growth and invasion, we searched for potential mRNA targets of miR-613 using the online bioinformatics TargetScan algorithm software. *SphK2* was predicted to be a target of miR-613 because of its positive effect on multiple cancer-related processes. To determine whether *SphK2* was negatively regulated by miR-613, the 3′-UTR of *SphK2* containing wild-type (WT) or mutant miR-613 target sequences was cloned into the psiCHECK-2 vector (Figure 4A). After cotransfection with miR-613 mimics, the luciferase activity of the WT 3′-UTR reporter gene significantly decreased, whereas the luciferase activity of the mutant reporter gene was not affected. These data suggested that miR-613 bound to the 3′-UTR of the *SphK2* gene (Figure 4B). We also found that *SphK2* expression was downregulated in TPC-1 cells transfected with miR-613 mimics compared with transfection with miR-C (Figure 4C). *SphK2* mRNA and protein levels were increased in BCPAP cells transfected with anti-miR-613 (Figure 4D).

**Figure 4:** *SphK2* is a direct target of miR-613 (**A**) Putative binding site ofmiR-613 in the *SphK2* 3′-UTR predicted by Target Scan. (**B**) Dual-luciferase activity of WT and mutant *SphK2* 3′-UTR reporter constructs in the presence of miR-613, relative to miR-C. (**C**) Expression of *SphK2* was detected in TPC-1 cells transfected with miR-613 mimics or miR-C using qRT-PCR and western blots. (**D**) Expression of *SphK2* was measured in BCPAP cells transfected with anti-miR-613 or anti-miR-C using qRT-PCR and western blots. (**E**) Expression of *SphK2* was examinedin PTC tissues (C) compared with non tumor tissues (N) by qRT-PCR. (**F**) Expression of *SphK2* was analyzed using immunohistochemistry.*P < 0.05.

We also examined the *SphK2* mRNA in 20 pairs of PTC tissue specimens and adjacent non tumor tissues. *SphK2* expression was higher in PTC specimens than corresponding non tumor thyroid tissues (Figure 4E). The inverse correlation between miR-613 and *SphK2* mRNA levels was further confirmed by Pearson correlation analysis in 20 PTC tissues (*r* = − 0.4480, *P* = 0.0476; Supplementary Figure S2). In addition, *SphK2* protein was analyzed using IHC on PTC tissues and nontumor tissues. The results showed that thirteen of 20 PTC samples (65%) exhibited positive *SphK2* staining in tumor cells, only 5% (1/20) of the nontumor thyroid tissues showed positive staining for *SphK2* (Supplementary Table S1), indicating that *SphK2* protein levels were significantly higher in PTC compared to normal tissues. We also studied the relationship between *SphK2* protein expression and clinicopathological data from 20 PTC patients and found a correlation between high *SphK2* expression levels and advanced clinical stage (*P* = 0.007) and classical papillary growth pattern (*P* = 0.042) (Supplementary Table S2).

### Restoration of SphK2 rescues tumor suppression by miR-613

To investigate whether the suppressive effects of miR-613 on the proliferation, migration and invasion of PTC cells was mediated by *SphK2* repression, we rescued *SphK2* expression in miR-613-overexpressing K1 and TPC-1 cells. *SphK2* restoration not only increased the proliferation of miR-613-transfected cells, but also partially increased their migration and invasion capacity compared with negative control cells (Figure 5). Importantly, TPC-1 cells transfected with *SphK2* expression vector partially reversed the inhibitory effect of miR-613 on tumor growth *in vivo* (Supplementary Figure S3). These results suggested that miR-613 suppressed PTC growth and metastasis by targeting *SphK2*.

**Figure 5:** Ectopic expression of *SphK2* restores the effects of miR-613 on cell proliferation, migration and invasion in PTC cells K1 and TPC-1 cells were respectively co-transfected with miR-613 and *SphK2* ORF without the 3′-UTR. (**A**) *SphK2* expression was measured using western blots for each group of transfected K1 and TPC-1 cells. (**B**–**D**) Cell proliferation by MTT assays, migration capacity by colony formation assays, and invasion capacity by transwell assays.*P < 0.05.

## DISCUSSION

MiRNAs regulate the expression of a variety of genes involved in cancer progression [20] and carcinogenesis [21, 22]. In this study, we observed that miR-613 was frequently downregulated in PTC cell lines and sample specimens, consistent with the findings of our preliminary study based on microarray analysis [14]. Functional analyses showed that overexpression of miR-613 suppressed cell proliferation, migration and invasion *in vitro* and inhibited tumor growth *in vivo*. *SphK2* was identified as a direct target of miR-613. *SphK2* expression was inversely correlated with miR-613 expression and rescuing *SphK2* expression reversed the suppressive effects of miR-613 on proliferation and invasion of PTC cells. Taken together, our work suggests that miR-613 exerts its suppressive effect on growth and metastasis of PTC by targeting *SphK2*.

Several miRNAs are reported to be abnormally expressed in PTC and involved in PTC pathogenesis. Liu *et al*. reported that mir-204-5p is downregulated in PTC tissues and functions as a potential tumor suppressor in PTC by targeting *IGFBP5* [23]. Huang *et al*. found that forced expression of miR-219-5p suppresses PTC cell proliferation and migration and promotes apoptosis [24]. Colamaio *et al*. showed that miR-191 is also downregulated in PTC [25]. In our recent study, miR-613 expression was significantly downregulated in PTC [14]. However, to date, studies on the biological function and molecular mechanism of miR-613 in PTC remain limited. Therefore, we selected miR-613 for further investigation in this study.

MiR-613 is reported to be downregulated in several types of cancer including prostate and ovarian cancer and esophageal squamous cell carcinoma [26–28]. In this study, we confirmed that miR-613 was downregulated in PTC. To better understand the function of miR-613 in PTC, the effect of miR-613 on PTC cell growth was examined *in vitro* using MTT and colony formation assays and *in vivo* using a xenograft tumor model. Overexpression of miR-613 significantly inhibited PTC cell proliferation *in vitro* and suppressed PTC tumor growth *in vivo*. Transwell assays suggested that overexpression of miR-613 inhibited the migratory and invasive ability of PTC cells. These results suggested that the ability of miR-613 to regulate cell growth, migration and invasion may contribute to PTC initiation and progression.

To further understand the mechanisms underlying the ability of miR-613 to inhibit cell growth, migration and invasion in PTC, we identified *Sphk2* as a potential target gene of miR-613 using bioinformatic analysis. Increasing evidence suggests that alterations in *SphK2* expression contribute to the pathogenesis of many human cancers [29–31]. *SphK2* overexpression in bladder cancer cells is closely implicated in tumor progression. Silencing of *SphK2* might inhibit the proliferation and migration of bladder cancer cells [29]. Knockdown of *SphK2* leads to decreased proliferation and enhanced chemosensitivity and apoptosis to gefitinib in non-small cell lung cancer [30]. The novel *SphK2* inhibitor ABC294640 induces growth inhibition and apoptosis in transformed and primary colorectal cancer cells, suggesting that *SphK2* may be involved in colorectal cancer development [31]. In this study, we found that *SphK2* was a target gene of miR-613 and restoration of *SphK2* expression abolished the inhibitory effect of miR-613 on cell proliferation and invasion. Inaddition, miR-613 expression was inversely correlated with *SphK2* expression in PTC tissues. Our study provides a new mechanism for *SphK2* regulation in PTC.

In summary, miR-613 regulated PTC cellular proliferation, migration, invasion and tumor growth by targeting *SphK2*. Our findings may help to further elucidate the molecular mechanisms underlying PTC progression and provide candidate targets for prevention and treatment of PTC.

## MATERIALS AND METHODS

### Patients and clinical tissue specimens

Samples of 20 pairs of primary PTC tissues and adjacent non tumor tissues were obtained from patients undergoing surgery at the Sixth People's Hospital Affiliated with Shanghai Jiao Tong University (Shanghai, China). The collection and use of patient samples was reviewed and approved by the Ethics Committee of the Sixth People's Hospital Affiliated with Shanghai Jiao Tong University, and written informed consent was obtained from each patient. Specimens were immediately snap-frozen in liquid nitrogen and stored at − 80°C until processing.

### Cell lines and cell culture

Human PTC cell lines (TPC-1, BCPAP, K1) and the human thyroid epithelial cell line Nthy-ori3-1 were purchased from the Cell Bank of the Chinese Academy of Sciences (Shanghai, China) and cultured in RPMI-1640 (Invitrogen, Carlsbad, CA, USA) supplemented with100 units/ml penicillin (Sigma-Aldrich, St. Louis, MO, USA), 0.1 mg/ml treptomycin (Enpromise, Hangzhou, China), and 10% fetal bovine serum. All cell lines were maintained in a humidified incubator of 5% CO_2 in air at 37°C._

### RNA isolation and quantitative real-time PCR analysis

RNA from cells or tissue samples was extracted using TRIzol reagent (Invitrogen). RNA was reverse transcribed to cDNA using Prime Script 1st Strand cDNA Synthesis Kit (TaKaRa, Dalian, China) according to the manufacturer's protocol. The cDNAs were subjected to qRT-PCR using SYBR Premix Ex Taq (TaKaRa) to detect miR-613 and SphK2 mRNA. U6 small nuclear or β-actin RNA were used as internal controls. Relative expression of target genes was determined using the 2^−ΔΔCt^ method.

### Oligonucleotides, plasmid construction and cell transfection

SphK2 coding sequences lacking the 3′-UTR were cloned into the pcDNA3.1 vector (Invitrogen) to generate the pcDNA3.1/SphK2 expression vector. Synthetic miR-613 mimics or control miRNA (miR-C) was used to transfect TPC-1 and K1 cells; a miR-613 inhibitor (anti-miR-613) or control miRNA (anti-miR-C) was used to transfect BCPAP cells. All synthetic miRNAs were from RiboBio (Guangzhou, China). Lipofectamine 2000 (Invitrogen) was used for all transfection experiments according to the manufacturer's instructions [32]. At 48 h after transfection, cells were harvested.

### Lentivirus production and transduction

miR-613 precursor sequences were amplified and cloned into the lentiviral vector pCDH-CMV-MCS-EF1-copGFP (System Biosciences, Mountain View, CA, USA). A lentiviral vector that expressed GFP alone was used as a control. The pCDH-miR-613 (Lv-miR-613) or pCDH-control (Lv-ctrl) vectors were cotransfected with the packaging plasmids psPAX2 and pMD into HEK 293T cells using Lipofectamine 2000 (Invitrogen). After 48 hours, virus particles were harvested.

### Cell proliferation and colony formation assays

Cell proliferation was evaluated by 3-(4,5-dimethyl-2-thiazolyl)-2,5-diphenyl-2H-tetrazolium bromide (MTT) assays. Cells were seeded into 96-well plates at 2000 cells per well and cultured for indicated times, followed by incubation at 5% CO_2_ and 37°C following the manufacturer's instructions. Results were measured as absorbance at 490 nm using a microplate reader absorbance test plate (Molecular Devices, Sunnyvale, CA, USA). Cells were detected for three wells per group. Colony formation ability was determined by plating at 300 cells per well into six-well plates and culturing for 12 days. Cells were fixed with methanol and stained with crystal violet. Stained colonies were imaged and counted.

### Cell migration and invasion assays

For invasion assays, chamber inserts were coated with Matrigel (BD Biosciences, San Jose, CA, USA). Cells were added to the upper chamber of Matrigel-coated inserts in 24-well plates and incubated for 24 h. Non invading cells were removed; cells attached to the bottom of the membrane were fixed with methanol, stained with crystal violet and counted under an inverted microscope. Transwell migration assays were performed as invasion assays, but without the Matrigel coating.

### Immunohistochemical staining analysis

Immunohistochemical (IHC) stainingwas performed as previously described using anti-SphK2((Santa Cruz Biotechnology, Santa Cruz, CA, USA) [29]. The degree of immunostaining of SphK1 proteins was scored by two observers blinded to clinical data. The intensity of immunoreactivity was classified as 0 (negative), 1 (weak, light yellow), 2 (moderate, yellow brown), or 3 (strong, brown). The proportion score was semiquantitative and graded as 0 (no positive tumor cells), 1 (< 10%), 2 (10–50%), or 3 (> 50%). These summed scores were calculated and divided into negative (0), weak (1–2), moderate (3), and strong (4–6) staining groups. For statistical purposes, the final scores of moderate and strong groups were considered as positive, and others were considered as negative.

### Western blotting

Protein extracted from cells using PIPA lysis buffer (Beyotime, Jiangsu, China) was measured with the bicinchoninic acid method (Pierce, Rockford, IL, USA). Equal amounts of protein were separated by 10% sodium dodecyl sulfatepolyacrylamide gel electrophoresis and transferred to polyvinylidene difluoride membranes. Membranes were incubated with primary antibody against *SphK2* (Santa Cruz Biotechnology) at 1:1000 dilution. Horseradish peroxidase-labeled secondary antibody was added, and specific protein signal bands were detected using an enhanced chemiluminescence detection reagent (Thermo Scientific, Rockford, IL, USA).

### *In vivo* tumorigenesis assays

For *in vivo* tumorigenesis assays, 1 × 10^6^ Lv-miR-613 or Lv-ctrl infected TPC-1 cells were subcutaneously injected into the flanks of female BALB/c-nude mice at 6–7 weeks of age. Tumor size was determined by measuring tumor length and width every three days. Tumor volume (mm^3^) was estimated using the formula: tumor volume = 0.5 × (length × width^2^). At 36 days after injection, animals were sacrificed and subcutaneous tumors were weighed. All animal handling and research protocols were approved by the Animal Care and Use Ethics Committee.

### Dual-luciferase assays

The 3′-UTR of SphK2 containing predicted miR-613 binding sites was amplified from human cDNA and cloned into the psiCHECK-2 dual-luciferase expression vector (Promega, Madison, WI, USA). Mutant 3′-UTR was obtained by overlap-extension PCR. K1 and TPC-1 cells were cotransfected with psiCHECK-SphK2-3′UTR-WT/MU and miR-613 using Lipofectamine 2000. Luciferase activity was measured with a dual-luciferase reporter assay system (Promega) at 48 h after transfection. Results were presented as the ratio of Renilla luciferase activity to firefly luciferase activity.

### Statistical analysis

All data were presented as mean ± standard deviation (SD) from at least three separate experiments. Differences between groups were analyzed using Student's *t*-test. SPSS 13.0 software (SPSS, Inc., Chicago, IL, USA) was used for statistical analysis. *P* values of 0.05 or less were considered statistically significant.

## SUPPLEMENTARY MATERIALS


